The article "Breast cancer screening: are we seeing the benefit?" was published in 2012. Journal: BMC Med.

# Breast cancer screening: are we seeing the benefit?

**DOI:** 10.1186/1741-7015-10-106

**Published:** 2012-09-20

**Authors:** Donella Puliti, Marco Zappa

**Affiliations:** 1 Clinical and Descriptive Epidemiology Unit, ISPO - Cancer Prevention and Research Institute, Via delle Oblate 2, 50141 Florence, Italy

**Keywords:** Mammography screening, breast cancer mortality, case-control studies, incidence-based mortality studies, analysis of trends

## Abstract

A decline in breast cancer mortality has been observed in western European Countries since the middle of the 1990s.

Different methodological approaches, including case-control studies, incidence-based mortality studies, and trend studies, have been used to assess the effectiveness of mammography screening programmes in reducing breast cancer mortality. However, not all methods succeed in distinguishing the relative contributions of service screening and taking correctly into consideration the potential source of bias that might affect the estimate.

Recently, a review of six case-control studies confirmed a breast cancer mortality reduction ranging from 38% to 70% among screened women. This figure is in accordance with the estimate obtained from incidence-based mortality studies if screening compliance is taken into account. We will describe the methodological constraints of mortality trend studies in predicting the impact of screening on mortality and the necessary caution that must be applied when interpreting the results of such studies.

In conclusion, when appropriate methodological approaches are used, it is evident that mammographic screening programmes have contributed substantially to the observed decline in breast cancer mortality.

## Introduction

Screening mammography is aimed at detecting breast cancer in an early stage in women without breast symptoms. The efficacy of mammography screening programmes has been assessed in eight randomized controlled trials conducted in Sweden, Scotland, New York, and Canada in the 1970s and 1980s [1]. In 2002 an International Agency for Research of Cancer (IARC) expert group has reached a consensus, based on review of published evidence, that mammographic screening is effective in reducing mortality from breast cancer [2]. A meta-analysis indicated a 30% reduction in breast cancer (BC) mortality among women aged 50 to 74 years [3]. In December 2003 the European Council recommended the implementation of mammographic screening in all the Member States. On these bases, mammographic screening programmes have been implemented in many European countries. The extension and timing of the implementation of population-based screening in the different countries were recently documented in the European Cancer Screening Report [4]. In 2007 about 54 million women in the age range 50 to 69 years in the European Union were targeted for breast cancer screening in the 22 Member States which had adopted policies aiming for implementation of population-based screening programmes.

Now that screening is widespread, non-randomized observational studies will become the main contributors of new information on the impact of breast cancer screening as a public health policy [5]. Different statistical methods including case-control studies [6,7], incidence-based mortality studies [8,9] and trend studies [10-12] have been used to assess the effectiveness of service screening. However, not all methods succeed in distinguishing the relative contributions of service screening and taking correctly into consideration the potential sources of bias that might affect the estimate. Following, we will discuss the main methodological approaches, highlighting their strengths and weaknesses.

## Case-control studies

The case-control study is a traditional tool for the evaluation of the effect of screening on BC mortality. This approach has also been used extensively for evaluating the efficacy of cervical and colorectal cancer screening [13,14].

The case-control study design has been used in several studies because of its efficiency. The rationale of these studies is the comparison of the screening histories in two groups of women, namely: (1) those who have died from breast cancer (cases); and (2) women sampled from the source population from which cases were drawn (controls). The collection of screening histories of a limited number of subjects allows a more accurate and valid evaluation than it could obtain for an entire population.

In 2010 a review of recent case-control studies on the effectiveness of population-based BC screening was carried out by Paap and colleagues [6]. Authors investigated the study design of six case-control studies [15-20] conducted in East Anglia (UK), Wales, Iceland, central and northern Italy, South Australia, and The Netherlands, and concluded that the design was quite similar. As shown in Table 1, the reduction of BC mortality in the different case-control studies ranged from 38% to 70% in the screened women compared with the unscreened women [15-20]. Analysis by exposure to screening measures the benefit of screening among women who agree to be screened, and therefore the result may be affected by self-selection bias. In all selected studies, a correction for self-selection bias was made using the method described by Duffy [21], and the corrected estimate was reported. Recently, a large case-control study [7] conducted in The Netherlands confirmed the beneficial effect of screening among women invited and participated in national mammography screening programme (OR = 0.51, 95%CI: 0.40-0.66).

**Table 1:** Design aspects and odds ratios (ORs) (crudes and corrected for self-selection bias) of six case-control studies.

Paper	Country	Time period of breast cancer deaths	Cases (*n*)	Screening exposure	Crude Ors (95% CI)	ORs adjusted for self-selection bias
Allgood *et al. *[15]	UK	1995-2004	284	Ever/Never attendance before (pseudo) diagnosis	0.35 (0.24-0.51)	0.52 (0.32-0.84)
Fielder *et al. *[16]	Wales	1998-2001	419	Ever/Never attendance before (pseudo) diagnosis	0.62 (0.47-0.82)	0.75 (0.49-1.14)
Gabe *et al. *[17]	Iceland	1990-2002	226	Ever/Never attendance before (pseudo) diagnosis	0.59 (0.41-0.84)	0.65 (0.39-1.09)
Paap *et al. *[18]	Netherlands	2004-2005	118	Screened at index invitation	0.30 (0.14-0.63)	0.24 (0.10-0.58)
Puliti *et al. *[19]	Italy	1988-2002	1750	Ever/Never attendance before (pseudo) diagnosis	0.46 (0.38-0.56)	0.55 (0.36-0.85)
Roder *et al. *[20]	Australia	2002-2005	491	Ever/Never attendance before (pseudo) diagnosis	0.59 (0.47-0.74)	0.70^a^

Source: Paap *et al.*, 2010 [11] modified.

^a^Values of confidence interval not reported in the paper.

The validity of case-control design for evaluating screening programmes has been largely discussed [22]. One of the main potential sources of bias is the so-called 'self-selection bias'. In other words screening participants and non-participants could present genuine differences of risk factors associated with dying from breast cancer. This reasoning is hypothetical and it is based on the argument 'we cannot exclude'. For example, screening participants may belong to a higher educational or socioeconomical status (SES). This status can be associated with a better access to quality treatment, so that we cannot exclude that the effect of the observed lower mortality is due to better treatment of higher SES. First of all it is worth mentioning that, as far as risk factors for BC are concerned, several studies have reported an inverse pattern: excesses in BC incidence in high female socioeconomic strata were seen in most populations [23,24]. Moreover we studied in depth the service mammographic screening programme in Florence, Italy. In this city a mammographic screening programme was implemented in the early 1990s. Recently [25] we documented that small differences in SES were observed among participants and no participants and that, after adjustment for SES and marital status, the decrease in BC mortality among screened women was in the range observed in case-control studies (RR = 0.55, 95%CI: 0.41-0.75 and RR = 0.49, 95%CI: 0.38-0.64 for the age groups 50-59 and 60-69 years, respectively). In other words the hypothesis that different SES played a major role in the observed decrease in mortality from BC is not confirmed.

## Incidence-based mortality

Incidence-based mortality (IBM) studies are those studies including only BC deaths occurring in women with BC diagnosed after their first invitation to screening. The IBM rate is different from the usual mortality rate because the population forms the denominator at diagnosis rather than at death [26]: person years at risk were counted from the date of first invitation until the date of death, emigration, or end of follow-up. All BC deaths among the cases diagnosed after the first invitation and until the end of follow-up were included in the numerator of the IBM rate.

The IBM rate in a population invited to screening was compared with the IBM rate expected without screening [9]. A key issue of these studies was thus how the BC mortality expected in the absence of screening was estimated. In the literature two different approaches were used: expected BC mortality was estimated from historical data adjusted for changes in breast cancer mortality over time [27]; or from a contemporaneous cohort of women not yet invited to screening [8]. In some cases both comparison groups were used [9]. It is worth noting that this intention-to-treat approach allows comparing invited and uninvited women, thus overcoming the self-selection bias.

Using this approach, the effect of screening is clearly evidenced and a reduction in BC mortality of around 25% was estimated [8,9,27]. This latter figure is in accordance with the above-mentioned results of case-control studies [6,7] if screening compliance is taken into account.

## Mortality temporal trends

Analysis of temporal trends in BC mortality rates is a tool frequently used due to the common availability of the data from population statistics and the apparent methodological easiness. Analyses were usually based on the comparison of BC mortality rates before and after the introduction of screening or on the comparison of the annual percentage change in BC mortality in areas with an active screening programme and in unscreened areas [10-12]. We will briefly describe the methodological constraints of temporal correlation studies in predicting the impact of screening on mortality, focusing on the necessary caution that must be applied when interpreting the results of such studies.

Analyses of temporal trends could be misleading due to multiple methodological failures. First, this type of study does not distinguish BC deaths in women who were diagnosed before the start of the screening programme from those diagnosed after the initiation of screening. It appears obvious that screening can only possibly have an effect on women not already diagnosed with BC. The correct way of performing statistical analyses is using the IBM method [26]. Second, the analyses could be misleading as they do not acknowledge that only a minority of women in the 'screened area' are actually screened; not all the women of the target population are invited to screening (for example during the implementation phase) and only a proportion of invited women are actually screened (according to compliance). To achieve a reliable assessment of the effect on mortality, it is necessary to make a direct link between a woman's BC death and her screening history.

Even if the comparison between screened and unscreened groups is set up properly, the interpretation of temporal mortality trend remains a very complex issue. It is well known that mortality rates are a function of both incidence and survival. Any changes of BC incidence rates over time will affect the cause-specific mortality rates in the subsequent years. The second determinant of the mortality rate, cancer survival, can be modified in two different ways: the advance of diagnosis and the improvement in therapy. All these factors (namely changes in incidence, stage at diagnosis, and therapeutic regimens) interact with each other to modify the mortality rates over time. The challenge is to assess the relative contribution of each factor to the reduction in BC mortality.

Recently, the effectiveness of mammography screening programmes in reducing BC mortality has been questioned on the basis of some observational studies analyzing mortality trends [10,11]. These analyze the temporal correlation between statistical aggregates: this approach weakens the evidence for a causative role of screening in changing mortality patterns. Moreover they compared very large and inhomogeneous areas. It is worth noting that an effect on mortality has been observed when comparing small areas in a more homogeneous situation. For example, comparing two areas of the province of Florence, where BC screening programmes started in the 1970s and in 1990s, it was showed that a mortality reduction of about 30% is attributable to screening in the early screening area [12].

## Conclusions

Given the methodological constraints of temporal correlation studies in predicting the impact of screening on mortality, the analysis of trends in BC mortality should be interpreted with caution. When specific studies evaluating the exposure to screening at an individual level are performed (including case-control studies and IBM studies), the effect of mammography screening on the reduction of BC mortality is evident and incontrovertible.

## Competing interests

The authors declare that they have no competing interests.

## Authors' contributions

PD and ZM conceived the scheme of the paper. PD wrote the manuscript and ZM revised it. Both authors approved the final manuscript.

## Authors' information

PD, statistician and master in Epidemiology, works at the Cancer Prevention and Research Institute (ISPO) since 2004 and she has been involved in several studies on breast, cervix, and colorectal cancer screening. ZM, medical doctor, is the director of the Italian National Centre of Screening Monitoring. He is the head of the Unit of Screening Evaluation at ISPO since 2004 and he is co-author of more than 200 peer-reviewed papers.

## Pre-publication history

The pre-publication history for this paper can be accessed here:

http://www.biomedcentral.com/1741-7015/10/106/prepub
